The article "A Higher-Order Galerkin Time Discretization and Numerical Comparisons for Two Models of HIV Infection" was published in 2022. Journal: Comput Math Methods Med.

# A Higher-Order Galerkin Time Discretization and Numerical Comparisons for Two Models of HIV Infection

**DOI:** 10.1155/2022/3599827

**Published:** 2022-11-09

**Authors:** Attaullah, Şuayip Yüzbaşı, Sultan Alyobi, Mansour F. Yassen, Wajaree Weera

**Affiliations:** ^1^Department of Mathematics and Statistics, Bacha Khan University Charsadda, KP 24461, Pakistan; ^2^Department of Mathematics, Faculty of Science, Akdeniz University, TR-07058 Antalya, Turkey; ^3^King Abdulaziz University, College of Science & Arts, Department of Mathematics, Rabigh, Saudi Arabia; ^4^Department of Mathematics, College of Science and Humanities in Al-Aflaj, Prince Sattam Bin Abdulaziz University, Al-Aflaj 11912, Saudi Arabia; ^5^Department of Mathematics, Faculty of Science, Damietta University, New Damietta, 34517 Damietta, Egypt; ^6^Department of Mathematics, Faculty of Science, Khon Kaen University, Khon Kaen 40002, Thailand

## Abstract

Human immunodeficiency virus (HIV) infection affects the immune system, particularly white blood cells known as CD4+ T-cells. HIV destroys CD4+ T-cells and significantly reduces a human's resistance to viral infectious diseases as well as severe bacterial infections, which can lead to certain illnesses. The HIV framework is defined as a system of nonlinear first-order ordinary differential equations, and the innovative Galerkin technique is used to approximate the solutions of the model. To validate the findings, solve the model employing the Runge-Kutta (RK) technique of order four. The findings of the suggested techniques are compared with the results obtained from conventional schemes such as MuHPM, MVIM, and HPM that exist in the literature. Furthermore, the simulations are performed with different time step sizes, and the accuracy is measured at various time intervals. The numerical computations clearly demonstrate that the Galerkin scheme, in contrast to the Runge-Kutta scheme, provides incredibly precise solutions at relatively large time step sizes. A comparison of the solutions reveals that the obtained results through the Galerkin scheme are in fairly good agreement with the RK4 scheme in a given time interval as compared to other conventional schemes. Moreover, having performed various numerical tests for assessing the efficiency and computational cost (in terms of time) of the suggested schemes, it is observed that the Galerkin scheme is noticeably slower than the Runge-Kutta scheme. On the other hand, this work is also concerned with the path tracking and damped oscillatory behaviour of the model with a variable supply rate for the generation of new CD4+ T-cells (based on viral load concentration) and the HIV infection incidence rate. Additionally, we investigate the influence of various physical characteristics by varying their values and analysing them using graphs. The investigations indicate that the lateral system ensured more accurate predictions than the previous model.

## 1. Introduction

Despite recent scientific advancements and substantial health-care initiatives, HIV/AIDS infection remains one of the most devastating diseases in human history. So still, several communities are still seriously impacted by this disease. At the moment, the global spread of HIV infection has an influence on the rising prevalence of other infectious diseases. Infectious diseases are illnesses that can be diagnosed clinically and have a large impact on the human community. They are caused by bacterial pathogens such as microorganisms, retroviruses, fungal, and parasitic agents or by harmful proteins known as prions. The most common are bacterial infectious diseases and tuberculosis, as well as virus-borne HIV and influenza [1, 2]. The hepatitis C virus (HCV) is highly widespread, with almost 71 million cases globally, and coinfections with HIV are also extremely frequent, with approximately 2.3 million coinfections [3]. Infection with HIV destroys the body's immune system; affects bodily organs such as the brain, kidney, and heart; and leads to death. Unfortunately, there is presently no treatment for this infectious illness. However, there are effective retroviral medications for improving patients' health complications. HIV is spread through sexual contact, sharing needles, and direct interaction with virus-infected blood or other bodily fluids, as well as mother-to-child transmission during delivery [2]. HIV is the virus that causes a disease known as immunodeficiency syndrome (AIDS), which weakens the body's capability to fight infection and leaves it vulnerable to attacks from contagious diseases. To improve health-care therapy, a detailed overview of the inflammatory and coagulation processes in HIV infection is essential [4]. In humans, CD4+ T-cells are HIV's targeted cells, and these cells play an essential role in the immune system's response. Their depletion can have a wide range of implications, potentially disrupting the immune system's functionality. Therefore, the reduction in the number of these cells is utilised as a symptomatic and illness stage indicator. In illnesses such as allergies and autoimmune disorders, regulatory T-cells (Treg) play significant roles in maintaining self-tolerance and immunological regulation. These cells also have a role in suppressing efficient immune responses to microbial organisms and cancerous cells [5]. Since the investigation is about the density of CD4+ T-cells, we will refer to T-cells and I-cells as healthy/infected CD4+ T-cells throughout the rest of the manuscript.

Numerous investigations have been conducted in order to identify the transmission dynamics of biological processes and infections. Cao et al. [6] presented a comprehensive approach to identifying successful treatment approaches and druggable targets by investigating regulatory interactions of cell phenotypic switching using precisely calculated probability landscapes of response networks. Mathematical formulation of infectious illnesses, such as HIV/AIDS coinfection and acute infection, is identified as a vital tool for understanding the dynamics of disease elimination and/or control [7]. The significance of immunological responses to HIV in modelling was highlighted by [8]. Omondi et al. [9] developed and evaluated a model containing a sex population that examined the HIV infection dynamics in both males and females. Vaidya et al. [10] examined how morphine affects resistivity to target cells, viral dynamics, and viral replication in a steady state, T-cell loss, and the efficiency of antiretroviral treatment (ART). They also looked into how morphine can boost basic reproduction rates, which poses significant challenges to HIV prevention. Vaidya et al. [11] established a viral infection model and investigated the role of antibody responses in reducing viral infection rates during infection. Calshaw and Raun [12] developed a model which consists of populations of T-cells, I-cells, and virus particles. Yusuf et al. [13] introduced a model and analysed the transmission behaviours of HIV infection. Singh [14] suggested a fractional order HIV model, with plasma densities of T-cells, I-cells, and free virus. They examined the dynamics of fractional HIV infection in T-cells as well as the impact of treatment. Thirumalai et al. [15] investigated the fractional order differential equations to analyse the combination of drug treatments for HIV infection. AlShamrani [16] suggested and evaluated an adaptive immune response model for HIV infection. Zaka Ullah and Baleanu [17] presented the SICA model in a fractional structure for the transmission dynamics of HIV/AIDS. Thirumalai et al. [18] studied HIV infection for T-cells using a model based on a system of differential equations. They evaluated and assessed an approximate solution of the mathematical model and presented a count of T-cells, I-cells, and viruses present at any given instant. Khan and Odinsyah [19] investigated HIV dynamics using a fractional operator of the Caputo type. They utilised the data of HIV infection cases in Indonesia from 2006 to 2018 to approximate the HIV model and determine the basic reproduction number. They proceeded by providing a mathematical description of the HIV/AIDS population. Chen and Zheng [20] explored the formation of spatial patterns in a predator-prey model with predator-taxis under homogenous zero-flux boundary conditions. They used the predator-taxis coefficient as the Turing bifurcation's possible critical value to play its part in constructing the spatial pattern. Chen and Wu [21] explored the diffusive nutrient-microorganism dynamics in a spatially heterogeneous environment. Chen et al. [22] studied the pattern formation and secondary instabilities of the Gierer-Meinhardt model, an activator-inhibitor system, including the Eckhaus instability and zigzag instability. By performing a linear stability analysis at the unique positive equilibrium, conditions on the Hopf bifurcation and Turing instability are discovered. Chen et al. [23] suggested a predator-prey model with a delayed ratio. They explored the system's Turing-Hopf bifurcation and established amplitude equations using the multiple time scale methodology. Theoretical and numerical simulations are used to find spatiotemporal solutions. Abdel et al. [24] examined the accurate travelling wave solutions of the fractional model of HIV-1 for T-cells and the effects of medication therapy. Naik et al. [25] suggested a Caputo-like fractional order model of HIV-1 that incorporates interactions between cancer cells and shows the chaotic behaviour. Raza et al. [26] developed a delayed model to study HIV dynamics in the community as well as the stability of a susceptible-infectious-immune system with a delay period.

In the literature, a variety of traditional analytical and numerical schemes are used to find the approximate solution of various models to describe the HIV dynamics. The homotopy analysis method (HAM) was applied by Ismail and Alomari [27], Ongun [28] performed the Laplace Adomian decomposition technique (LADM), Doğan [29] implemented the multistep LADM, and Yüzbaşı and Karaçayır [30] developed a novel computational approach based on exponential polynomials related to the Galerkin scheme for the HIV infection model. Recently, Sohaib [31] have studied the Legendre wavelet collocation method and the continuous Galerkin-Petrov scheme to obtain the solutions to the HIV model. They made comparison of the outcomes and highlighted the precision and efficacy of the proposed schemes in contrast to other approaches employed to the model. Yüzbaşı et al. [32] presented an exponential approach for numerical solutions to the HIV model based on T-cells. The technique involves exponential polynomials and collocation points. Haq et al. [33] investigated the dynamics of a fractional order smoking cessation model and presented an approximate solution based on the Laplace transformation. Attaullah et al. [34] have applied the Galerkin time discretization scheme to the following HIV models and compared the results with the Runge-Kutta method. Yüzbaşı [35] developed the Bessel collocation approach and implemented it on the HIV T-cell model. The suggested technique comprises of resolving the problem to the system of nonlinear algebraic equations by expanding the approximate solutions with unknown coefficients employing Bessel polynomials. For the numerical investigation, Ahmed et al. [36] proposed an extended temporal model of HIV with medication treatment impact using the backward Euler and Crank-Nicolson techniques. The HIV model of T-cells was explored by Yüzbaşı [37], and an operational technique was suggested to numerically address the model problem. Merdan [38] utilised the homotopy perturbation method (HPM) to examine the numerical outcomes of HIV model. Attaullah [39] approximates the solution of the HIV infection model with full logistic proliferation and variable source terms employing the Galerkin scheme. The modified multivariational iteration method (MVIM) is used by Merdan et al. [40] in order to approximate the suggested model. Multistage homotopy perturbation method (MuHPM) is used by Leal et al. [41] and demonstrated the path tracking behaviour of HIV dynamics.

### 1.1. Fundamental Objectives

The fundamental aim of the present paper is to examine the well-known HIV infection model of T-cells characterized by Leal et al. [41] based on three coupled nonlinear ordinary differential equations. The mentioned model is solved by applying the Galerkin discretization scheme known as the continuous Galerkin-Petrov method, briefly cGP(2) method. This method has superiority to some extent over the other traditional techniques. Each time interval in the cGP(2) method has two unknowns that can be computed by solving a 2 × 2 block system. The suggested approach is accurate to three orders over the whole time period and even demonstrates super convergence to four orders in discrete time points. To illustrate the reliability of the Galerkin scheme, the model is solved using the Runge-Kutta technique of order four, shortened as the RK4 method. Our second aim is to compare the solutions of the Galerkin method with the findings of other techniques, e.g., MuHPM [42], MVIM [40], and HPM [38]. All the findings are visualised through different graphs. The comparative study was performed to validate the accuracy and computational cost (in terms of time) of the Galerkin and RK4 methods for the same and different time step sizes. Therefore, to having an idea about the accuracy and reliability of the approximate solutions obtained from the proposed technique, the well-known classical RK4 method is also implemented. Estimate the absolute errors between the results of both schemes to better understand and authenticate our proposed method's applicability in practical problems. The assessment of the absolute values of errors between the Galerkin scheme and RK4 scheme solutions shows that the solutions provided are more accurate in comparison to the solutions obtained through conventional schemes. The graphical and tabular outcomes demonstrated that the proposed scheme is very accurate and achieves highly accurate results at a larger step size in comparison to the existing techniques employed for the mentioned model. The Galerkin scheme is an adaptive scheme that achieves the same accuracy at a larger step size at a lower cost. The detailed analysis of the aforementioned model demonstrates that the Galerkin scheme is more authentic and accurate than the previous approaches employed for the model. Our third aim is to develop it by the insertion of a new dynamic supply term dependent on the viral density for the generation of new T-cells and a mass action term in the HIV model. Leal et al. [41] suggested the HIV infection model with a stable parameter for the production of new T-cells from the thymus. However, HIV has the potential to invade T-cells in the thymus, which might affect the generation of new cells from the thymus. Therefore, the model discussed in [41] is extended by introducing a variable source term (“*s*(*V*) = 0.5*ℑs* + (*sℑ*/*ℑ* + *V*)” discussed in [43, 44]) based on viral density. In addition, the mass action term *kVT* is introduce to explain how infection occurs when the virus interacts with T-cells, causing free virus to be eradicated at a rate of −*kVT*, where *k* indicates the infection rate. Moreover, the variation of different clinical parameters involved in the model is observed by changing their values. A computer program written in mathematical software is used to perform these computations.

### 1.2. The Outline of the Paper

The rest of the article is structured as follows: Section 4 introduces the fundamental formulation of the HIV model.  Section 3.1 provides the Galerkin method implemented for the model. Numerical results, behaviours of different parameters, and comparison of the solutions of the Galerkin method and RK4 method with other classical techniques applied to the model are discussed in Section 4.1.  Section 5 gives the conclusion and summary of the article.

## 2. Basic Mathematical Structure of the HIV Infection Model

This section concerns the model suggested by Leal et al. [41]. Our first aim in this study is to apply the continuous Galerkin-Petrov time discretization scheme [31, 34] to the following HIV model and to compare outcomes with the methods existing in literature to validate the accuracy and efficiency of the scheme and the MATLAB code. The model is as follows:

(1) $$\begin{array}{c} \frac{dT}{dt}=s-\mu_{T}T+rT\left(1-\frac{T+I}{T_{\max}}\right),\\ \frac{dI}{dt}=kVT-\mu_{I}I,\\ \frac{dV}{dt}=N\mu_{I}I-\mu_{V}V+kVT, \end{array}$$

where the state variables *T*(*t*), *I*(*t*), and *V*(*t*) show the density of T-cells, I-cells, and the HIV virus in the blood, respectively. The diagrammatic illustration of the HIV model and the structure of the HIV virus are given in Figure 1. The initial conditions of state variables, different parameters, and constants with their explanations are provided in Table 1.

## 3. The Numerical Schemes

This section discusses the numerical schemes used to solve the above-mentioned model. Nowadays, the Galerkin approach has been used effectively to handle a wide range of complicated problems in engineering and science, seen for example [31, 45–49]. We implemented the technique on the HIV model discussed in [41]. In addition, we employ the conventional Runge-Kutta approach to assess the precision of the Galerkin scheme findings.

### 3.1. The Continuous Galerkin-Petrov (cGP) Technique

The system of ODE's for the considered model can be written follows:

Find $\tilde{u}:\left[0,t_{\max}\right]⟶V={\mathbb{R}}^{d}$ like as follows:

(2) $$\begin{array}{c} \begin{array}{c} d_{t}\tilde{u}\left(t\right)=F\left(t,\tilde{u}\left(t\right)\right)\forall t\in I,\\ \tilde{u}\left(0\right)=u_{0}, \end{array} \end{array}$$

where *d*_*t*_ shows the time derivative of $\tilde{u}\left(t\right)$, *ℐ* = [0, *T*] is the total interval, and $\tilde{u}\left(t\right)=\left({\tilde{u}}_{1}\left(t\right),{\tilde{u}}_{2}\left(t\right),{\tilde{u}}_{3}\left(t\right)\right)\in V\Rightarrow \tilde{u}\left(0\right)=\left({\tilde{u}}_{1}\left(0\right),{\tilde{u}}_{2}\left(0\right),{\tilde{u}}_{3}\left(0\right)\right)\in V$ are the initial values of $\tilde{u}\left(t\right)$ at *t* = 0. We also assume that $\left({\tilde{u}}_{1}\left(t\right),{\tilde{u}}_{2}\left(t\right),{\tilde{u}}_{3}\left(t\right)\right)=\left(T\left(t\right),I\left(t\right),V\left(t\right)\right)$ which implies that $\left({\tilde{u}}_{1}\left(0\right),{\tilde{u}}_{2}\left(0\right),{\tilde{u}}_{3}\left(0\right)\right)=\left(T\left(0\right),I\left(0\right),V\left(0\right)\right)$. The function *ℱ* = (*f*_1_, *f*_2_, *f*_3_) is nonlinear and is described as *ℱ* : *ℐ* × *𝒦*⟶*𝒦*.

The *weak formulation* (see [31, 34, 45–49] for explanations) of a the problem (2) is follows: find $\tilde{u}\in X$ such that $\tilde{u}\left(0\right)={\tilde{u}}_{0}$ and

(3) $$\begin{array}{c} \int_{I}\langle d_{t}\tilde{u}\left(t\right),v\left(t\right)\rangle dt=\int_{I}\langle F\left(t,\tilde{u}\left(t\right),\nu \left(t\right)\right)\rangle dt\text{ for all }\nu \in Y, \end{array}$$

where *𝒳* and *𝒴* represent the solution and test space, respectively, to explain the time discretization of a variational type problem (2).

To characterize the function $t⟶\tilde{u}\left(t\right)$, we describe the space *C*(*ℐ*, *𝒦*) = *C*^0^(*ℐ*, *𝒦*) that is the space of continuous functions $\tilde{u}$: *ℐ*⟶*𝒦* equipped with the norm as follows:

(4) $$\begin{array}{c} {\left\|\tilde{u}\right\|}_{C\left(I,K\right)}=\underset{t\in I}{\sup}{\left\|\tilde{u}\right\|}_{K}. \end{array}$$

We will use the space *L*^2^(*ℐ*, *𝒦*) as the space of discontinuous functions which is given by

(5) $$\begin{array}{c} L^{2}\left(I,K\right)=\left\{\tilde{u}:I⟶K:{\left\|\tilde{u}\right\|}_{L^{2}\left(I,K\right)}={\left(\int_{I}{\left\|\tilde{u}\right\|}_{K}^{2}dt<\infty \right)}^{1/2}\right\}. \end{array}$$

In time discretization, we split the intervals *ℐ* into *N* subintervals *ℐ*_*τ*_ = [*t*_*τ*−1_, *t*_*τ*_], where *τ* = 1, ⋯, *N* and 0 = *t*_0_ < *t*_1_ < *t*_2_ < ⋯<*t*_*N*−1_ < *t*_*N*_ = *T*. The parameter *j* indicates the time discretization parameter, as well as the maximum time step size $j=\underset{1\leq \tau \leq N}{\max}j_{\tau }$, where *j*_*τ*_ = *t*_*τ*_ − *t*_*τ*−1_ is the length of *n*th time interval *ℐ*_*τ*_. The following set of time intervals *M*_*j*_ = {*ℐ*_1_, ⋯, *ℐ*_*N*_} will be called the time mesh. We find out the solution $\tilde{u}$: *ℐ*⟶*𝒦* on each time interval *ℐ*_*τ*_ by a function ${\tilde{u}}_{j}$: *ℐ*⟶*𝒦* which is a piecewise polynomial of some order *l* w.rt time. The time-discrete solution space for ${\tilde{u}}_{j}$ is *𝒳*_*j*_^*l*^ ⊂ *𝒳* and is defined by

(6) $$\begin{array}{c} X_{j}^{l}=\left\{\tilde{u}\in C\left(I,K\right){\left.:\tilde{u}\right|}_{I_{\tau }}\in {\mathbb{P}}_{l}\left(I_{\tau },K\right)\text{ for all }I_{\tau }\in {\text{M}}_{j}\right\}, \end{array}$$

where

(7) $$\begin{array}{c} {\mathbb{P}}_{l}\left(I_{\tau },K\right)=\left\{\tilde{u}:I_{\tau }⟶K:\tilde{u}\left(t\right)=\overset{l}{\underset{s=0}{\sum }}U^{s}t^{s},\text{for }all\;t\in I_{\tau },U^{s}\in K,\forall s\right\}. \end{array}$$

The discrete test space for ${\tilde{u}}_{ȷ}$ is *𝒴*_*ȷ*_^*l*^ ⊂ *𝒴* and is defined by

(8) $$\begin{array}{c} Y_{j}^{k}=\left\{v\in L^{2}\left(I,K\right)\text{: }{\left.v\right|}_{I_{\tau }}\in {\mathbb{P}}_{k-1}\left(I,K\right)\forall I_{\tau }\in M_{j}\right\}, \end{array}$$

which is composed of *l* − 1 piecewise polynomials (see [31, 34, 45–49] for details) and is discontinuous at the time step end nodes. We multiply equation (2) by the test function *ν*_*ȷ*_ ∈ *𝒴*_*ȷ*_^*k*^ and integrate over the interval *ℐ*. We get the discrete-time problem: find ${\tilde{u}}_{ȷ}\in {𝒳}_{ȷ}^{k}$ such that ${\tilde{u}}_{ȷ}\left(0\right)=0$ and

(9) $$\begin{array}{c} \int_{I}\langle {\tilde{u}}_{ȷ}^{\prime }\left(t\right),\nu_{ȷ}\left(t\right)\rangle dt=\int_{I}\langle F\left(t,{\tilde{u}}_{ȷ}\left(t\right),\nu_{ȷ}\left(t\right)\right)\rangle dt\forall \nu_{ȷ}\in Y_{ȷ}^{l}, \end{array}$$

where 〈·and·〉 represent the usual inner product in *L*^2^(*ℐ*, *𝒦*). This discretization is known as the exact *continuous* Galerkin-Petrov method or simply the “exact cGP(l) scheme” of order *k*. The Galerkin-Petrov name is due to the fact that the solution space *𝒳*_*ȷ*_^*l*^ is different from the test space *𝒴*_*ȷ*_^*l*^. The term “exact” denotes that the time integral on the right-hand side of equation (9) is determined exactly. Because the discrete test space *𝒴*_*ȷ*_^*l*^ is discontinuous, equation (9) could be computed by a time marching technique in which local problems on the interval are handled successively. Therefore, we select the test function *ν*_*ȷ*_(*t*) = *νφ*(*t*) with arbitrary time independent *ν* ∈ *𝒦* and a scalar function *φ* : *ℐ*⟶ℝ which is zero on *ℐ*|_*ℐ*_*τ*__ and a polynomial of order less than or equal to *l* − 1 on the time interval *ℐ*_*τ*_ = [*t*_*τ*−1_, *t*_*τ*_]. Then, we get from (9) the *ℐ*_*τ*_ problem of the exact cGP scheme of order *l*: find ${\left.{\tilde{u}}_{ȷ}\right|}_{{ℐ}_{\tau }}\in {\mathbb{P}}_{l}\left({ℐ}_{\tau },𝒦\right)$ such that

(10) $$\begin{array}{c} \int_{I_{\tau }}\langle d_{t}{\tilde{u}}_{ȷ}\left(t\right),\nu \rangle \varphi \left(t\right)dt=\int_{I_{\tau }}\langle F\left(t,{\tilde{u}}_{ȷ}\left(t\right)\right),\nu \rangle \varphi \left(t\right)dt\forall \nu \in K\forall \varphi \in {\mathbb{P}}_{l-1}\left(I_{\tau }\right), \end{array}$$

with the initial condition ${\tilde{u}}_{ȷ}{\left|{}_{{ℐ}_{\tau }}\left(t_{\tau -1}\right)={\tilde{u}}_{ȷ}\right|}_{{ℐ}_{\tau -1}}\left(t_{\tau -1}\right)$ for *τ* ≥ 2 and ${\left.{\tilde{u}}_{ȷ}\right|}_{{ℐ}_{\tau }}\left(t_{\tau -1}\right)={\tilde{u}}_{0}$ for *τ* = 1.

In case of a nonlinear function *ℱ*〈·, ·〉, we need to calculate the integrals numerically on the right-hand side of equation (10). The (*l* + 1)-point Gau*β*-Lobatto formula is exact if the function to be integrated has a polynomial of degree less than or equal to 2*l* − 1. As a result, this formula is applied to the integral on the left-hand side of (10) which will give the exact value. Then, the “*ℐ*_*τ*_ problem of the numerically integrated cGP(*l*) method” is as follows: find ${\left.{\tilde{u}}_{ȷ}\right|}_{{ℐ}_{\tau }}\in {\mathbb{P}}_{l}\left({ℐ}_{\tau },𝒦\right)$ such that ${\tilde{u}}_{ȷ}\left(t_{\tau -1}\right)={\tilde{u}}_{\tau -1}$,

(11) $$\begin{array}{c} \overset{l}{\underset{s=0}{\sum }}{\hat{w}}_{s}d_{t}{\tilde{u}}_{ȷ}\left(t_{\tau ,s}\right)\varphi \left(t_{\tau ,s}\right)=\overset{k}{\underset{s=0}{\sum }}{\hat{w}}_{s}F\left(t_{\tau ,s},{\tilde{u}}_{ȷ}\left(t_{\tau ,s}\right)\right)\varphi \left(t_{\tau ,s}\right)\forall \varphi \in {\mathbb{P}}_{l-1}\left(I_{\tau }\right), \end{array}$$

where *w*_*s*_ are the weights and $\hat{t}\in \left[-1,1\right],s=0,1,2,3,\cdots ,l$ represent the nodes on the reference interval. To find ${\tilde{u}}_{ȷ}$ on each time interval *ℐ*_*τ*_, we use a polynomial ansatz to illustrate it as follows:

(12) $$\begin{array}{c} {\tilde{u}}_{ȷ}\left(t\right)=\overset{k}{\underset{s=0}{\sum }}U_{\tau }^{s}\phi_{\tau ,s}\left(t\right)\forall t\in I_{\tau }, \end{array}$$

where the coefficients *U*_*τ*_^*s*^ are the components of *𝒦* and the functions *ϕ*_*τ*,*s*_ ∈ *ℙ*_*l*_(*ℐ*_*τ*_) are the Lagrange basis functions (see [31, 34, 45–49] for more details) with respect to *l* + 1 suitable nodal points *t*_*τ*,*s*_ ∈ *ℐ*_*τ*_ satisfying conditions mentioned below:

(13) $$\begin{array}{c} \phi_{\tau ,s}\left(t_{\tau ,r}\right)=\delta_{r,s},r,s=0,1,2,\cdots ,l, \end{array}$$

where *δ*_*r*,*s*_ is the Kronecker delta that is defined as

(14) $$\begin{array}{c} \delta_{r,s}=\left\{\begin{array}{cc} 1 & \text{if }r=s,\\ 0 & \text{if }r\neq s. \end{array}\right. \end{array}$$

Like in [50], the *t*_*τ*,*s*_ have been defined as the quadrature points of (*l* + 1)-point Gau*β*-Lobatto formula (for detail information, see [31, 34, 45–49]) on the interval *ℐ*_*τ*_. For the selection of initial conditions, we can set *t*_*τ*,0_ = *t*_*τ*−1_ which denotes the initial condition for equation (10)

(15) $$\begin{array}{c} \begin{array}{c} {\left.U_{\tau }^{0}={\tilde{u}}_{ȷ}\right|}_{I_{\tau -1}}\text{ if }\tau \geq 2,\\ \text{for }\tau =1\Rightarrow U_{\tau }^{0}={\tilde{u}}_{0}. \end{array} \end{array}$$

We define the basis functions *ϕ*_*τ*,*s*_ ∈ *ℙ*_*l*_(*ℐ*_*τ*_) via the affine reference transformation (see [31, 34, 45–49] for detail explanations) $\bar{T}:\hat{ℐ}⟶{ℐ}_{\tau }$, where $\hat{ℐ}=\left[-1,1\right]$ and

(16) $$\begin{array}{c} t=\bar{T}\left(\hat{t}\right)=\frac{t_{\tau }+t_{\tau -1}}{2}+\frac{{ȷ}_{\tau }}{2}\hat{t}\in I_{\tau }\forall \hat{t}\in I_{\tau },\tau =1,2,3\cdots ,N. \end{array}$$

Let $\hat{\phi_{s}}\in {\mathbb{P}}_{l}\left(\hat{ℐ}\right)$, *s* = 0, 1, ⋯, *l*, demonstrate the basis functions that meet the requirements

(17) $$\begin{array}{c} {\hat{\phi }}_{s}\left({\hat{t}}_{r}\right)=\delta_{r,s},\;r,s=0,1,\cdots ,l, \end{array}$$

where ${\hat{t}}_{0}=-1$ and ${\hat{t}}_{r}$, *r* = 1, 2, ⋯, *l*, are the quadrature points for the reference interval $\hat{ℐ}$. Then, we define the basis functions on the given interval *ℐ*_*τ*_ by the mapping

(18) $$\begin{array}{c} \phi_{\tau ,s}\left(t\right)=\hat{\phi_{s}}\left(\hat{t}\right)\text{ with }\hat{t}={\bar{T}}_{\tau }^{-1}\left(t\right)=\frac{2}{{ȷ}_{\tau }}\left(t+\frac{t_{\tau -1}-t_{\tau }}{2}\right)\in \hat{I}. \end{array}$$

Likewise, the test basis functions *φ*_*τ*,*r*_ are described by the suitable reference basis functions $\hat{\varphi }\in {\mathbb{P}}_{l-1}\left(\hat{ℐ}\right)$, i.e.,

(19) $$\begin{array}{c} \varphi_{\tau ,r}\left(t\right)=\hat{\varphi_{r}}\left({\bar{T}}_{\tau }^{-1}\left(t\right)\right)\;\forall t\in I_{\tau },r=1,2,\cdots ,l. \end{array}$$

From the representation (12), we get for $d_{t}{\tilde{u}}_{ȷ}$

(20) $$\begin{array}{c} d_{t}{\tilde{u}}_{ȷ}\left(t\right)=\overset{k}{\underset{s=0}{\sum }}U_{\tau }^{s}\phi_{\tau ,s}^{\prime }\left(t\right)\forall t\in I_{\tau }. \end{array}$$

By putting (20) in (10), we get

(21) $$\begin{array}{c} \int_{I_{\tau }}\langle d_{t}{\tilde{u}}_{ȷ}\left(t\right),\nu \rangle \varphi \left(t\right)\;dt=\int_{I_{\tau }}\langle \overset{l}{\underset{s=0}{\sum }}U_{\tau }^{s},\nu \rangle \phi_{s}^{\prime }\left(t\right)\varphi \left(t\right). \end{array}$$

The integral is now transformed into the reference interval *hatI* and computed using the (*l* + 1)-point Gau*β*-Lobatto quadrature formula which leads, for each test basis function *φ* ∈ *ℙ*_*l*−1_ and for all *ν* ∈ *𝒦*,

(22) $$\begin{array}{c} \int_{{\hat{I}}_{\tau }}\overset{l}{\underset{s=0}{\sum }}\langle U_{\tau }^{s},\nu \rangle {\hat{\phi }}_{s}^{\prime }\left(\hat{t}\right)\hat{\varphi }\left(\hat{t}\right)d\hat{t}=\int_{{\hat{I}}_{\tau }}\langle F\left(\omega_{\tau }\left(\hat{t}\right),\overset{l}{\underset{s=0}{\sum }}U_{\tau }^{s}\left(\hat{t}\right)\right),\nu \rangle \hat{\varphi }\left(\hat{t}\right)d\hat{t}\forall \nu \in K,\Rightarrow \overset{l}{\underset{\mu =0}{\sum }}{\hat{w}}_{\mu }\overset{l}{\underset{s=0}{\sum }}\langle U_{\tau }^{s},\nu \rangle {\hat{\phi }}_{s}^{\prime }\left({\hat{t}}_{\mu }\right)\hat{\varphi }\left({\hat{t}}_{\mu }\right)=\overset{l}{\underset{\mu =0}{\sum }}{\hat{w}}_{\mu }\langle F\left(\omega_{\tau }\left({\hat{t}}_{\mu }\right),\overset{l}{\underset{s=0}{\sum }}U_{\tau }^{s}{\hat{\phi }}_{s}\left({\hat{t}}_{\mu }\right)\right),\nu \rangle \hat{\varphi }\left({\hat{t}}_{\mu }\right), \end{array}$$

where ${\hat{w}}_{\mu }$ are the weights and ${\hat{t}}_{\mu }\in \left[-1,1\right]$ are the points of integration with ${\hat{t}}_{0}=-1$ and ${\hat{t}}_{l}=1$. If we choose the test functions *φ*_*τ*,*i*_ ∈ *ℙ*_*l*−1_(*ℐ*_*τ*_) such that

(23) $$\begin{array}{c} \hat{\varphi }\left(\hat{t_{\mu }}\right)={\left(\overset{\wedge }{w}\right)}^{-1}\delta_{r,\mu }\;r,\mu =1,2,\cdots ,l. \end{array}$$

Now find the coefficients that are unknown *U*_*τ*_^*s*^ ∈ *𝒦* for *s* = 1, ⋯, *l*,

(24) $$\begin{array}{c} \overset{l}{\underset{s=0}{\sum }}\alpha_{r,s}U_{\tau }^{s}=\frac{{ȷ}_{\tau }}{2}\left\{F\left(t_{\tau ,r},U_{\tau }^{s}\right)+\beta_{r}F\left(t_{\tau ,0},U_{\tau }^{s}\right)\right\}\forall i=1,2,\cdots ,l, \end{array}$$

where *U*_*τ*_^*s*^ = *U*_*τ*−1_^*s*^ for *τ* > 1 and $U_{1}^{0}={\tilde{u}}_{0}$ for *τ* = 1 and

(25) $$\begin{array}{c} \alpha_{r,s}={\hat{\phi }}_{s}^{\prime }\left({\hat{t}}_{r}\right)+\beta_{r}{\hat{\phi }}_{s}^{\prime }\left(t_{0}\right),\;\beta_{r}={\hat{w}}_{0}{\hat{\varphi }}_{r}\left({\hat{t}}_{0}\right). \end{array}$$

We will discuss the cGP(k) method for the cases *l* = 1 and *l* = 2 in the following subsections.

#### 3.1.1. The cGP(1) Method

We used the two point Gau*β*-Lobatto formula with *t*_*τ*,0_ = *t*_*τ*−1_, *t*_*τ*,1_ = *t*_*τ*_ and weights ${\hat{w}}_{0}={\hat{w}}_{1}=1$ which gives the well-known trapezoidal rule. We obtain *α*_1,0_ = −1, *α*_1,1_ = 1, and *β*_1_ = 1. For the single coefficient $U_{\tau }^{1}={\tilde{u}}_{ȷ}\left(t_{\tau }\right)\in 𝒦$, the problem leads to the following block equation:

(26) $$\begin{array}{c} \alpha_{1,1}U_{\tau }^{1}-\alpha_{\tau ,0}U_{\tau }^{0}=\frac{{ȷ}_{\tau }}{2}\left\{F\left(t_{\tau },U_{\tau }^{1}\right)+F\left(t_{\tau -1},U_{\tau }^{0}\right)\right\}. \end{array}$$

#### 3.1.2. The cGP(2) Method

Three-point Gau*β*-Lobatto formula (Simpson's rule) is used to define the quadratic basis functions with weights ${\hat{w}}_{0}={\hat{w}}_{2}=1/3$, ${\hat{w}}_{1}=4/3$, ${\hat{t}}_{0}=-1$, ${\hat{t}}_{1}=0$, and ${\hat{t}}_{2}=1$. Then, we get

(27) $$\begin{array}{c} \alpha_{r,s}=\left(\begin{array}{ccc} -\frac{5}{4} & 1 & \frac{1}{4}\\ 2 & -4 & 2 \end{array}\right),\\ \;\beta_{r}=\left(\begin{array}{c} \frac{1}{2}\\ -1 \end{array}\right),\\ r=1,2,\;s=0,1,2. \end{array}$$

Thus, the system to be solved for **U**_*τ*_^1^, **U**_*τ*_^2^ ∈ *𝒦* from the known **U**_*τ*_^0^ = **U**_*τ*−1_^2^ becomes

(28) $$\begin{array}{c} \alpha_{1,1}U_{\tau }^{2}=-\alpha_{1,0}U_{\tau }^{0}+{ȷ}_{2}^{\tau }\left\{F\left(t_{\tau ,1},U_{\tau }^{1}\right)+\beta_{1}F\left(t_{\tau ,0},U_{\tau }^{0}\right)\right\},\\ \alpha_{2,1}U_{\tau }^{1}+\alpha_{2,2}U_{\tau }^{2}=-\alpha_{2,0}U_{\tau }^{0}+\frac{{ȷ}_{\tau }}{2}\left\{F\left(t_{\tau ,2},U_{\tau }^{2}\right)+\beta_{2}F\left(t_{\tau ,0},U_{\tau }^{0}\right)\right\}, \end{array}$$

where **U**_*τ*_^0^ indicate the initial condition at the current time interval.

### 3.2. Runge-Kutta Method

This is a well-known technique of order four, established by Kutta [51] and extensively utilised for initial value problems (see [52, 53] for more details).

### 3.3. Comparison and Computation Analysis

This section demonstrates the significance of the Galerkin and RK4 methods to the system of ODE's 4.1–4.3 in the aforementioned model. The initial conditions and parameter values are given in Table 1. In order to determine the effectiveness of the suggested technique, we contrasted the numerical and graphical solutions achieved by the Galerkin scheme with those obtained by the RK4 method and other conventional methods, i.e., MuHPM [41], MVIM [40], and HPM [38], provided in Tables 2–4 for *T*(*t*), *I*(*t*), and *V*(*t*). After the evaluation, it was revealed that the proposed approach produced more precise findings than the solutions obtained through conventional approaches. Furthermore, numerical computations are carried out using the Galerkin scheme and the RK4 scheme with the same and different time step sizes. The absolute errors between the outcomes were assessed using both approaches, as demonstrated in Tables 5 and 6. From comparison, it is clearly visible that the Galerkin scheme achieves more precise findings at a larger step size as compared to the RK4 technique.  Figure 2 shows the results of both methods for *t* ∈ [0, 1] and *t* ∈ [0, 70] with *ȷ* = 0.1 steps. The figures showed that the results overlapped over each other throughout the time period. In addition, the analysis of the numerical costs for different step sizes in terms of time shows that the Galerkin method is more time-consuming as in comparison to the RK4 method is presented in Table 7 and Figure 3(f). The polar and bar graphs illustrate the absolute errors between the solutions of the Galerkin and RK4 approaches depicted in Figure 4. The mesh graphs for the solutions of the Galerkin method, RK4 method, MuHPM [41], MVIM [40], and HPM [38] are visualised in 3. Overall, we may conclude that the numerical approach reported in this article can be relied on to produce reasonably flexible and accurate results when applied to comparable problems.

## 4. Mathematical Formulation of the HIV Infection Model

The study of HIV/AIDS infection requires an understanding of T-cell population dynamics because T-cells are the major target of HIV particles. Since these cells are generated in the bone marrow, premature T-cells are directed to the thymus for further differentiation and maturation before becoming immune-competent T-cells. However, HIV may be able to infect these cells in both bone marrow and the thymus and destroy the supply of new cells [54]. But majority of the HIV models in the literature assumed with the constant rate of generation of new T-cells from the thymus. Herein, we modified the HIV model assumed by Leal et al. [41]. We consider the innovative model with the assumption that the production of new cells from the thymus is a decreasing function based on viral load (“*s*(*V*) = 0.5*ℑs* + (*sℑ*/*ℑ* + *V*)” used in [43, 44, 55]) rather than the constant source term. Further, include mass action term “*kVT*,” where *k* is the infection rate. Infection occurs when a virus infects T-cells, reducing them at the rate of “−*kVT*” and producing virus at the rate of “*kVT*.” It is observed that the mentioned model gives more accurate and realistic-based findings for T-cells, I-cells, and HIV. The new model is follows:

(29) $$\begin{array}{c} \frac{dT}{dt}=0.5Is+\frac{sI}{I+V}-\mu_{T}T+rT\left(1-\frac{T+I}{T_{\max}}\right)-kVT,\\ \frac{dI}{dt}=kVT-\mu_{I}I,\\ \frac{dV}{dt}=N\mu_{I}I-\mu_{V}V+kVT, \end{array}$$

where *T*(*t*), *I*(*t*), and *V*(*t*) represent the density of T-cells, I-cells, and virus particles in the blood, respectively. The diagrammatic illustration of the HIV model and the structure of the HIV virus are illustrated in Figure 1. Following confirmation of the aforementioned scheme and validation of the MATLAB code, we applied the aforesaid scheme to a novel established model and visualised the dynamical behaviour of the model with the interaction of major clinical parameters. The initial conditions of state variables, various parameters, and constants with their explanations are provided in Table 1 and *ℑ* = 1 mm^−3^.

### 4.1. Analysis and Discussions

In this section of the research, several numerical simulations are carried to illustrate the detailed behaviour of the proposed model. Figures 5(a)–5(c) depict that by increasing the quantity of free virus produced by reduction of T-cells, the concentration of T-cells increases at top level initially. But after ten days approximately, its wavelength starts decreasing with time and touches the lowest level. Due to killing of viral particles and cell response, the density of T-cells increases again after initial decline. However, immune cells are directly impacted by viral particles; their number steadily diminishes over time, indicating that T-cells are targeted by viruses. The increasing value of “*N*” gives rapid rise to the depletion of T-cells at huge level and is more predictable sign for AIDS. The profile of I-cells shows oscillatory behaviour, and the wavelength is increasing by increasing the generation rate of free virus “*N*.” The viruses attack the immunity cells and convert these T-cells into I-cells. Due to such virus replication and infection of T-cells, the amount of I-cells increases. Meanwhile, the immune system has the capability to identify viruses and destroy them to control the infection. Therefore, the rate of I-cells again decreases after seventy days approximately. The influence of growth rate (“*r*”) of the T-cell population on the dynamical behaviour of sate variables (*T*(*t*), *I*(*t*)*V*(*t*)) is visualised in Figures 5(d)–5(f). From the graphical view, it could be observed that state variables show considerably the same dynamics by increasing the growth rate and death rate but speeds up the decaying oscillation. The impact of increasing the death rate (*μ*_*T*_) of the T-cell population on the dynamical behaviour of sate variables is depicted in Figures 6(a)–6(c). If the mortality rate of T-cells increases, there is no significant influence on the density of T-cells in the earliest stages. Since the virus attacks T-cells on a continuous basis, a gradual but significant decline occurs after seventy days. Similarly, the time period for the concentration of I-cells and free HIV virus particles is affected slightly. Figures 6(d)–6(f) demonstrate that if the mortality rate of the I-cell population grows, the rate of T-cells reaches a maximum in the early days but begins to drop in concentration with the passage of time, and a continuous pattern of crest and trough with a small wavelength in density of T-cells could be noticed. The population of I-cells diminishes, although time has a vital effect, as seen in the graphs. Since HIV particles are latently present, they affect the number of I-cells, and their patterns display the same behaviour as I-cells. The infection rate oscillates over a seventy-day time-frame, and the death rate of I-cells has a significant effect on the growth of viral particles. By reducing the mortality rate of virus particles, the concentration of T-cells decreases with time, whereas speeding the depletion with longer wavelengths, as illustrated in Figure 7(a). The HIV particles target T-cells; their concentration rises if the mortality rate of HIV particles is lowered. Also, at the end of ten days, the initial and final densities of T-cells are almost identical, whereas the density of I-cells and viral particles grows and the time for growth in I-cell and viral particles decreases, as shown in Figures 7(b) and 7(c).

The phase and chaotic behaviour of the specified model are shown in Figures 7(d)–8(b). Many scientific and engineering applications are based on a system's chaotic nature [34]. It is well acknowledged that there is a substantial tendency toward understanding and representing chaotic system behaviours. The chaotic diagrams demonstrate the feasibility and application of the suggested numerical approach, which may be generalized to novel chaotic systems.

## 5. Concluding Remarks

In this paper, the continuous Galerkin-Petrov time discretization scheme is implemented for the model for HIV infection, which is comprised of three nonlinear ordinary differential equations. Afterwards, implement the RK4 method for solving the model and compare the solutions of both techniques. Moreover, a comprehensive analysis of the outcomes of the Galerkin method and RK4 method with findings of other schemes available in the literature is presented in detail. The assessment of the absolute values of errors between the Galerkin scheme and RK4 scheme solutions shows that the solutions provided are more accurate in comparison to the solutions obtained through conventional schemes. The graphical and tabular outcomes demonstrated that the proposed scheme is very accurate and achieves highly accurate results at a larger step size in comparison to the existing techniques employed for the mentioned model. The Galerkin scheme is an adaptive scheme that achieves the same accuracy at a larger step size at a lower cost. In comparison towards other approaches, our technique yields more accurate results than other methods that have addressed the same problem. The findings demonstrate that the approach employed may be utilised for numerous types of nonlinear systems of differential equations. The performance of the proposed approach demonstrates that these methods are logically effective and reliable for solving nonlinear problems in complex dynamical systems. On the other hand, we examined the dynamical behaviour of the model with a variable supply rate (depending on viral load) of new T-cells. The influence of significant clinical parameters on the dynamics of T-cells, I-cells, and free HIV virus particles is described and observed by varying their values. The main findings are as follows:

1. Increasing the density virus produced by per I-cells (*N*) increases the concentration of T-cells, I-cells, and virus particles
2. The decaying oscillatory behaviour is observed in the density of state variables by rising the value of *r*
3. By enhancing the mortality of I-cells, the density of T-cells and virus rises while the population of I-cells diminishes
4. The increase in population of all state variables is observed by decreasing the mortality rate of HIV

In addition, the phase and chaotic behaviour of the aforementioned model are presented. Many scientific and technical applications are predicated on the chaotic character of a system. It is widely accepted that there is a heavy tendency toward comprehending and portraying chaotic system behaviours. The chaotic diagrams show the practicality and accessibility of the suggested numerical technique, which may be expanded to novel chaotic systems.

In the future, we plan to elaborate on the research by incorporating vaccination rates and investigating their impact on the model's dynamical behaviour.

## Figures and Tables

**Figure 1:** The diagrammatic description of the model and HIV virus.

**Figure 2:** The geometrical comparison between the findings of the Galerkin and RK4 schemes for *T*(*t*), *I*(*t*), and *V*(*t*) for *t* ∈ [0, 70] and *t* ∈ [0, 1] with *j* = 0.1.

**Figure 3:** The mesh graphs of the Galerkin method, RK4 method, MuHPM [41], MVIM [40], and HPM [38] for the model and the computation cost in terms of CPU time (f).

**Figure 4:** The polar and bar graphs of errors between the findings of the Galerkin and RK4 schemes and bar graphs for the Galerkin and RK4 schemes for *T*(*t*), *I*(*t*), and *V*(*t*).

**Figure 5:** The impact of significant parameters on the HIV infection model for T-cell generation with varying source term (dependent on viral load).

**Figure 6:** The impact of significant parameters on the HIV infection model for T-cell generation with varying source term (dependent on viral load).

**Figure 7:** The impact of significant parameters on the HIV infection model for T-cell generation with varying source term (dependent on viral load) and phase diagram.

**Figure 8:** The phase diagram of HIV infection model including T-cell generation with varying source term (dependent on viral load).

**Table 1:** Description of state variables, parameters, and their values [41] (units: day^−1^ mm^−3^).

	Descriptions	Values
Dependent variables		
*T*_0_	Population of T-cells	0.10
*I*_0_	Population of I-cells	0.0
*V*_0_	Population of HIV particles	0.10

Parameters and constants		
*s*	The supply rate of T-cells	0.1
*r*	The growth rate of the T-cell population	3
*μ*_*T*_	The killing rate of T-cells	0.02
*μ*_*I*_	The killing rate of I-cells	0.3
*μ*_*V*_	The destruction rate of free virus	2.4
*k*	The infection rate of T-cells by free virus	2.4 × 10^−5^
*N*	The density of virus released by I-cells	Varies
*T*_max_	The maximum density of T-cells	1500

**Table 2:** The findings of the Galerkin method, RK4 method, MuHPM [41], MVIM [40], and HPM [38] for *T*(*t*).

*t*_*i*_	MuHPM [41]	MVIM [40]	HPM [38]	RK4 method	Present solutions
0.0	0.10000000	0.10000000	0.100000000	0.1000000000000	0.1000000000000
0.1	0.14635895	0.14635910	0.146358900	0.1463563334215	0.1463584928222
0.2	0.20880772	0.20880810	0.208799100	0.2088006788767	0.2088064964841
0.4	0.40623923	0.40624080	0.405606600	0.4062136749646	0.4062347843124
0.6	0.76442034	0.76442870	0.756448500	0.7643508145370	0.7644082444391
0.8	1.41403830	1.41409400	1.364215000	1.4138702489163	1.4140090611266
1.0	2.59157570	2.59192100	2.378679000	2.5911951903662	2.5915094589373
1.2	4.72392418	4.72578300	4.006512000	4.7230983734038	4.7237803350162
1.4	8.57832730	8.58722300	6.521303000	8.5765895980001	8.5780243166268
1.6	15.5227925	15.5616700	10.27357000	15.519228130625	15.522170203755
1.8	27.9613543	28.1196100	15.70079000	27.954219776306	27.960106298377
2.0	50.0080707	50.6147700	23.33740000	49.994185112927	50.005637473626
3.0	605.328400	758.304100	121.4166000	605.19715873002	605.30962600425
4.0	1387.07811	-38782.630	428.1830000	1387.0365698936	1387.0734647790
5.0	1484.41661	-1.2822*E*+7	1179.633000	1484.4129741128	1484.4162185194
10	578.768500	-7.535*E*+18	31121.36000	578.01860976666	578.80322177533
30	42.9620000	-7.954*E*+65	6710438.000	42.988262407096	42.979478181920
70	51.1260000	-8.86*E*+159	4.49161*E*+08	50.731613644543	50.729213455592

**Table 3:** The findings of the Galerkin method, RK4 method, MuHPM [41], MVIM [40], and HPM [38] for *I*(*t*).

*t*_*i*_	MuHPM [41]	MVIM [40]	HPM [38]	RK4 method	Present solutions
0.0	0.00000000	0.00000000	0.00000000	0.0000000000000	0.0000000000000
0.1	0.00000286	0.00000286	0.00000286	0.0000028645332	0.0000028648471
0.2	0.00000603	0.00000603	0.00000603	0.0000060318789	0.0000060325464
0.4	0.00001316	0.00001315	0.00001315	0.0000131564860	0.0000131579785
0.6	0.00002122	0.00002122	0.00002122	0.0000212206776	0.0000212231597
0.8	0.00003018	0.00003017	0.00002994	0.0000301728102	0.0000301764661
1.0	0.00004004	0.00004002	0.00003918	0.0000400314158	0.0000400364581
1.2	0.00005088	0.00005084	0.00004844	0.0000508700174	0.0000508766963
1.4	0.00006283	0.00006270	0.00005697	0.0000628162070	0.0000628248219
1.6	0.00007608	0.00007574	0.00006354	0.0000760684228	0.0000760793421
1.8	0.00009096	0.00009011	0.00006649	0.0000909418517	0.0000909555499
2.0	0.00010799	0.00010597	0.00006346	0.0001079686795	0.0001079858141
3.0	0.00030568	0.00021559	-0.0001816	0.0003055957917	0.0003056674148
4.0	0.00210920	0.00040533	-0.0014837	0.0021084186444	0.0021090778379
5.0	0.02011931	0.00074045	-0.0055038	0.0201107695276	0.0201179825874
10.0	828.594800	0.01387534	-0.2285212	828.38422383941	828.56686684266
30.0	775.293700	1625.28280	-64.142730	775.29918583941	775.28577475039
70.0	594.704000	2.2292*E*+13	-4621.4330	594.00643606878	594.00643962536

**Table 4:** The findings of the Galerkin method, RK4 method, MuHPM [41], MVIM [40], and HPM [38] for *V*(*t*).

*t*_*i*_	MuHPM [41]	MVIM [40]	HPM [38]	RK4 method	Present solutions
0.0	0.10000000	0.10000000	0.10000000	0.1000000000000	0.1000000000000
0.1	0.07866315	0.07866318	0.07866315	0.0786638145502	0.0786632635595
0.2	0.06187980	0.06187991	0.06187825	0.0618808474016	0.0618799805166
0.4	0.03829484	0.03829596	0.03819947	0.0382961304371	0.0382950575829
0.6	0.02370450	0.02371029	0.02268158	0.0237057031284	0.0237047074676
0.8	0.01468033	0.01470042	0.00925511	0.0146813143229	0.0146804932549
1.0	0.00910082	0.00915723	-0.0104847	0.0091015790768	0.0091009447531
1.2	0.00565326	0.00579375	-0.0498259	0.0056538216298	0.0056533518393
1.4	0.00352541	0.00385124	-0.1294878	0.0035258155248	0.0035254781828
1.6	0.00221475	0.00293882	-0.2801688	0.0022150382652	0.0022148022419
1.8	0.00141046	0.00297863	-0.5450945	0.0014106541633	0.0014104933204
2.0	0.00092039	0.00426490	-0.9825656	0.0009205205645	0.0009204146275
3.0	0.00032941	0.13649810	-9.1749200	0.0003293651184	0.0003293983282
4.0	0.00141090	5.40689000	-43.553080	0.0014103809499	0.0014108255861
5.0	0.01292825	214.291400	-143.65180	0.0129227583497	0.0129273975037
10.0	668.789590	2.095*E*+10	-5456.7680	668.57158158359	668.75792981167
30.0	983.982000	1.916*E*+42	-150636600	983.92573498469	983.92438186017
70.0	769.490000	1.602*E*+106	-1.0827*E*+8	768.96288598031	768.95708309906

**Table 5:** The absolute errors between the findings of the Galerkin and RK4 schemes for *T*(*t*), *I*(*t*), and *V*(*t*) with same step size and *t* ∈ [0, 70].

|*cGP*(2)_*j*=0.01_ − *RK*4_*j*=0.01_|			
*t*_*i*_	*T*(*t*)	*I*(*t*)	*V*(*t*)
0.0	0.00000000000000*E*-10	0.00000000000000*E*-14	0.00000000000000*E*-11
0.1	2.84775258929670*E*-10	3.46123001238724*E*-14	4.45784936742299*E*-11
0.2	7.67201135953854*E*-10	7.50830062186403*E*-14	7.01317059981221*E*-11
0.3	1.55009055591293*E*-09	1.21598593011158*E*-13	8.27457546925814*E*-11
0.4	2.78372330742016*E*-09	1.74456149260862*E*-13	8.67752675270950*E*-11
0.5	4.68632355143939*E*-09	2.34046319786763*E*-13	8.53053669369608*E*-11
0.6	7.57295037789874*E*-09	3.00841803183537*E*-13	8.04949266963728*E*-11
0.7	1.18961085426861*E*-08	3.75390284178614*E*-13	7.38314721859812*E*-11
0.8	1.83025996580710*E*-08	4.58311269117091*E*-13	6.63192608468810*E*-11
0.9	2.77127207848338*E*-08	5.50296584017097*E*-13	5.86177772987639*E*-11
1.2	8.98785703640215*E*-08	8.88763672032833*E*-13	3.77432252118837*E*-11
1.4	1.89002486550294*E*-07	1.17644883093106*E*-12	2.69146562675848*E*-11
1.6	3.87287119707480*E*-07	1.52607589651126*E*-12	1.85752377021564*E*-11
1.8	7.73954734967219*E*-07	1.95361702347036*E*-12	1.23150862337690*E*-11
2.0	1.50285070077416*E*-06	2.48521210934657*E*-12	7.65154150976499*E*-12
3.0	1.44064168807745*E*-05	1.06163661303844*E*-11	6.34902492992889*E*-12
4.0	4.45008413407777*E*-06	9.61197484453114*E*-11	6.36393082328879*E*-11
5.0	3.44141881214455*E*-07	1.02496256620954*E*-09	6.58341856724087*E*-10
10	2.90578410613307*E*-05	2.45547904569321*E*-05	2.57475288663045*E*-05
30	1.43229695481750*E*-06	2.60882575275900*E*-06	5.73396846448304*E*-07
70	4.48719525536490*E*-07	1.54975691657455*E*-06	1.31251681523281*E*-06

**Table 6:** The absolute errors for *T*(*t*), *I*(*t*), and *V*(*t*) between the Galerkin and RK4 techniques for *t* ∈ [0, 70] with different step sizes.

|*cGP*(2)_*j*=0.01_ − *RK*4_*j*=0.0001_|			
*t*_*i*_	*T*(*t*)	*I*(*t*)	*V*(*t*)
0.0	0.00000000000000*E*-11	0.00000000000000*E*-15	0.00000000000000*E*-12
0.1	5.86432846727547*E*-11	7.12909557572966*E*-15	8.69847249784783*E*-12
0.2	1.57959229030169*E*-10	1.54760669814828*E*-14	1.36827840724330*E*-11
0.3	3.19075987853523*E*-10	2.50826784472732*E*-14	1.61410537713458*E*-11
0.4	5.72855207714440*E*-10	3.60121817349207*E*-14	1.69235597757833*E*-11
0.5	9.64069601927520*E*-10	4.83457641053866*E*-14	1.66324766459613*E*-11
0.6	1.55727908346393*E*-09	6.21799635977353*E*-14	1.56892346336868*E*-11
0.7	2.44506304092340*E*-09	7.76247081478616*E*-14	1.43842576738606*E*-11
0.8	3.75948450148655*E*-09	9.48020382628059*E*-14	1.29135296206284*E*-11
0.9	5.68795943678424*E*-09	1.13844887293310*E*-13	1.14057773642484*E*-11
1.0	8.49506598399330*E*-09	1.34896515615809*E*-13	9.94224494399454*E*-12
1.2	1.83776105444622*E*-08	1.83649035106863*E*-13	7.31735158576718*E*-12
1.4	3.84712617318428*E*-08	2.42403387401731*E*-13	5.19390173231438*E*-12
1.6	7.82565194867857*E*-08	3.12689110715247*E*-13	3.55596108114753*E*-12
1.8	1.54546054176308*E*-07	3.96344591803606*E*-13	2.32396979264748*E*-12
2.0	2.94468271988535*E*-07	4.95918884842010*E*-13	1.40495156741166*E*-12
3.0	2.23191591430805*E*-06	1.76651054895061*E*-12	1.14225539834048*E*-12
4.0	5.47712943443912*E*-07	1.65905887118678*E*-11	1.07716444271155*E*-11
5.0	4.52982931165025*E*-08	1.77432183529058*E*-10	1.13838096935104*E*-10
10	4.84750069063011*E*-06	4.06695653509814*E*-06	4.55263102594472*E*-06
30	2.30107175980265*E*-07	4.45262458015350*E*-07	1.09476786747109*E*-07
70	7.22985902257278*E*-08	2.61271452473011*E*-07	2.25629946726258*E*-07

**Table 7:** The numerical cost in terms of the CPU time (in seconds) for the cGP(2) scheme and RK4 scheme for *t* ∈ [0, 70].

CPU time (in seconds)		
1/*j*	cGP(2) method	RK4 method
70	0.851371	0.058463
100	0.958954	0.054076
200	1.607708	0.067753
500	2.687663	0.084981
1000	4.473871	0.124775
1500	5.245537	0.199593
2000	6.021062	0.234840
5000	10.244101	0.515386
10000	17.510589	0.859149
20000	31.660067	1.945279

## Data Availability

All the data are available in the manuscript.
